The article "Road-Type Classification with Deep AutoEncoder" was published in 2023. Journal: Comput Intell Neurosci.

# Road-Type Classification with Deep AutoEncoder

**DOI:** 10.1155/2023/1456971

**Published:** 2023-03-14

**Authors:** Mohale E. Molefe, Jules R. Tapamo

**Affiliations:** School of Engineering, University of KwaZulu Natal, Durban, South Africa

## Abstract

Machine learning algorithms are among the driving forces towards the success of intelligent road network systems design. Such algorithms allow for the design of systems that provide safe road usage, efficient infrastructure, and traffic flow management. One such application of machine learning in intelligent road networks is classifying different road network types that provide useful traffic information to road users. We propose a deep autoencoder model for representation learning to classify road network types. Each road segment node is represented as a feature vector. Unlike existing graph embedding methods that perform road segment embedding using the neighbouring road segments, the proposed method performs embedding directly on the road segment vectors. The proposed method performs embedding directly on the road segment vectors. Comparison with state-of-the-art graph embedding methods show that the proposed method outperforms graph convolution networks, GraphSAGE-MEAN, graph attention networks, and graph isomorphism network methods, and it achieves similar performance to GraphSAGE-MAXPOOL.

## 1. Introduction

Throughout the world, the number of vehicles and road users is increasing, and this has created traffic problems such as traffic congestion, accidents, and fuel cost. The rise of such traffic problems has led to the need to design and develop smart cities. Smart city design integrates physical, digital, and human systems in the built environment to facilitate the planning, construction, and management of the city's infrastructure [1]. Smart cities cover a wide range of applications within the transport and health industries. One key element of smart city design within the transport industry is the intelligent road network system design, which aims to ensure efficient traffic flow by minimising traffic problems. Intelligent road networks have also seen a wide range of applications in the domain of autonomous vehicles.

The use of intelligent road networks system is widely accepted in many countries, and its use is not only limited to traffic flow control and information but also expands to efficient infrastructure and road safety usage. Machine learning algorithms have been the driving force behind the successes of intelligent road networks; indeed, access to big data has opened doors to the development of various intelligent road network models. One such application of machine learning in road networks is classifying different road types. Road-type classification models are becoming important, as they can be embedded in interactive maps to provide helpful traffic information to road users. Other benefits of road-type classification include efficient traffic flow management, avoidance of congested routes, avoidance of routes where accidents are likely to occur, avoidance of routes with many intersections, and model integration to autonomous vehicles.

The article "Road-Type Classification with Deep AutoEncoder" was published in 2023. Journal: Comput Intell Neurosci.

However, modelling road networks with machine learning is complex due to the lack of available feature extraction methods for representing road-types as feature vectors. Thus, researchers have introduced deep learning embedding methods to learn the spatial information of road networks to automatically extract features in the network data. These embedding methods are termed graph representation learning (GRL) as they rely on the spatial connection of different objects within the road network structure; thus, each object's feature vectors are constructed by leveraging its spatial connection with neighbouring objects. The main goal of GRL methods is to achieve automatic feature extraction on the non-Euclidean graph data space without relying on the actual object attributes.

In this work, however, a method for representing different road types as feature vectors is proposed, such that machine learning classification algorithms can be trained and evaluated on these features. We take full advantage of the state-of-the-art baseline road network feature extraction method proposed in [2]. Furthermore, we introduce a deep autoencoder (DAE) embedding method to reduce the dimensions of feature vectors obtained by the baseline method. We then pass the feature vectors extracted by our DAE method to several machine learning classification algorithms; we select the classifier with the highest performance measure.

The rest of the paper is organised as follows. In Section 2, we present the literature study and related works.  Section 3 provides the materials and methods used to build our model. In Section 4, we present the experimental results obtained by the proposed method, and we further compare the results to some of the state-of-the-art methods found in the literature. Finally, in Section 5, we conclude our work and provide recommendations for future work.

## 2. Background and Related Work

Graph theory is the fittest paradigm for modelling road networks, as it embraces all the topological information of any road network. Apart from the spatial road networks, graphs diagrammatically represent all transport networks, including highway, transits networks, air, and water. Thus, attributes such as speed, travel times, number of lanes, and head ways can be represented. A network's topological spatial structure is represented by graphs composed of lines and points. Lines are also called edges, while points are nodes or vertices. Therefore, graphs can represent the topology and spatial structure of a road network such that nodes represent intersections, dead-ends, and locations of interest on the roads, while edges represent the road segments between such nodes.

The article "Road-Type Classification with Deep AutoEncoder" was published in 2023. Journal: Comput Intell Neurosci.

Machine learning in road networks has had many successes in facilitating important traffic information such as traffic forecasting [3–5], speed limit annotation [6–8], and travel time estimation [9–11]. However, machine learning in road networks for modelling road-type classification is often challenging due to a lack of attributes representing different road types. Thus, it sounds reasonable to apply deep learning methods to automatically learn the network's structure and represent every road segment by aggregating its neighbouring road segments. However, solving a learning problem on graphs is challenging. This is because many widely used data types, such as images and texts, are not structured as graphs. Also, the underlying connectivity patterns on the graph-structured data are more complex and non-Euclidean.

The fundamental solution to modelling complex, non-Euclidean patterns is to learn the graph representation from a low-dimensional Euclidean space using the GRL methods. Once the low-dimensional representations are learned, graphs-related problems such as node and link predictions can be achieved. Also known as graph embedding functions, the main goal of the GRL methods is to pack the properties of every road segment into a vector with a smaller dimension; this enables road segment similarity in the original complex graph space to be quantified in the embedded feature space using standard metrics. Several embedding methods have been proposed in the literature for modelling road networks. In [12], a hybrid graph convolution neural network (HGCN) method is proposed for traffic flow prediction in highway networks, where nodes represent the toll stations while edges represent road segments between two toll stations. In addition to modelling the spatial feature of the highway, the authors achieved better traffic flow prediction by considering factors such as time, space, weather conditions, and data type of each toll station.

It is worth noting that the HGCN method proposed in [12] uses local neighbourhood aggregation to learn the spatial connection of toll stations, and it cannot integrate road segment features into the learning process. This is valid since many state-of-the-art GRL methods rely on node features only. However, road segment features in road networks not only provide the connectivity information of two nodes but can also provide important, descriptive information that could be significant for the learning representation. To tackle this problem, the notion of relational fusion networks (RFN) is proposed in [13], for the speed limit classification and estimation tasks. RFN integrates edge information on the representation learning using the novel graph convolution operator. The RFN operator aggregates information over the relations between nodes instead of aggregating the information over neighbouring nodes.

The article "Road-Type Classification with Deep AutoEncoder" was published in 2023. Journal: Comput Intell Neurosci.

To the best of our knowledge, the work proposed in [2] is the only available work in the literature that classifies different road types on a graph dataset extracted from Open Street Maps (OSMnx). Similar to RFN, the authors used the dual graph generated by the line graph transformation of the original graph to incorporate the edge features into the learning process. Thereafter, a method for generating road segment features is proposed based on information such as the length of the road segment, speed limit, and midpoint coordinates of the adjacent start and end nodes. The authors further compared the performance of learning representation using several embedding methods, including graph convolution networks (GCN) [14], GraphSAGE [15], graph attention networks (GAT) [16], and graph isomorphism network (GIN) [17] in inductive and transductive tasks, and in supervised and unsupervised learning tasks. In addition, a new GRL method, graph attention isomorphism network (GAIN), is proposed.

In our work, we attempt to improve the robustness of road segment features extracted in [2], by using the deep autoencoder (DAE) model as the embedding function; furthermore, we focus on the transductive and supervised learning settings only since these are the settings that achieved the highest accuracy in [2]. Unlike most graph embedding methods proposed in the literature, our DAE model does not construct the vector representation of the target road segment by aggregating over its neighbouring segments; instead, it operates directly on the high dimensional feature vectors of each road segment and produces compact feature vectors in a much smaller dimensional space. We then pass these compact features into several machine learning algorithms and report the results using the microaveraged *f*1-score. Finally, we compare our highest f1-score to the f1-score obtained using the methods proposed in [2].

## 3. Materials and Methods

As depicted in Figure 1, our proposed method for road-type classification comprises 6 steps. First, we extract the original road network graph dataset of Linkoping city from OSMnx. Edges in the original graph represent the road segments, while nodes represent information such as intersections and crossroads. In the second step, we transform the original graph into a line graph representing road segments as nodes. In the third step, we use the original and transformed graphs to derive attributes and represent every road segment as a feature vector. To the best of our knowledge, steps 1 to 3 of our proposed method follow a similar procedure proposed in [2]. In step 4, we introduce the deep autoencoder model as the embedding function, and dimensionality reduction is performed. In step 5, we use the feature vectors obtained by our embedding function to train, validate, and test the deep neural networks, support vector machines, and K-nearest neighbor classifiers. We then select the classifier with the highest microaveraged *f*1-score and compare our obtained results to some of the state-of-the-art embedding methods for solving a similar task to ours.

The article "Road-Type Classification with Deep AutoEncoder" was published in 2023. Journal: Comput Intell Neurosci.

### 3.1. Input Dataset

Similar to the transductive setting in [2], the input dataset used to conduct the experiments in our work is the road network graph dataset of Linkoping city. The dataset was extracted from OSMnx within a 14 km radius of the city centroid. The obtained graph dataset is represented as *G*=(*V*, *E*), where *V* and *E* are set of nodes and set edges, respectively. Edges represent road segments, and nodes represent crossroads, intersections, and junctions. Some of the preprocessing steps on the obtained graph involved transforming *G* into an undirected graph, consolidating parallel edges, and intersections within a 10 m distance.

### 3.2. Line Graph Transformation

As depicted in Figure 2, the original graph *G* is converted to line graph *L*(*G*), such that edges (road segments) in *G* become nodes in *L*(*G*) and two edges (two road segments) that share a node (intersection) in *G* become an edge in *L*(*G*). Transforming *G* to *L*(*G*) has two significant advantages. Firstly, graph embedding methods in the literature are designed for nodes and not edges; thus, the transformed graph *L*(*G*) has road segments as nodes. Secondly, nodes (cross-roads, intersections, and junctions) on the original graph do not have the essential information required for road-type classification tasks.  Algorithm 1 gives the steps used to transform *G* to *L*(*G*).

### 3.3. Class Distribution

Road segments in OSMnx are tagged with their corresponding road-type labels, thus allowing for a supervised classification task to be accomplished. However, 15 road-type labels are obtained, and some of these labels rarely occur on our obtained dataset. Therefore, the distribution of data is highly characterised by extreme class imbalances. To tackle this problem, we follow the same technique as in [2], where the authors merged and relabelled road types as shown in Table 1.

The article "Road-Type Classification with Deep AutoEncoder" was published in 2023. Journal: Comput Intell Neurosci.

### 3.4. Feature Engineering

Feature generation of each road segment is conducted by extracting its descriptive attributes from the edges of the original graph and nodes of the transformed graph. Indeed, attributes such as the width, length, number of lanes, and speed limit of light vehicles and heavy vehicles provide useful road segment information required for feature generation. Nevertheless, we generate the road segment feature vectors using four main components as in [2] to compare the results fairly. As shown in Table 2, these four components yield a 58-dimensional feature vector for every road segment.

Let *l* represent the road segment length, (*x*, *y*) be the midpoint coordinates of two nodes in longitude and latitude directions, respectively, and *S*={*s*_1_, *s*_2_, *s*_3_,…, *s*_*m*_} be the one hot encoding vector of *m* speed limits. Then, the final feature vector of each road segment is generated using Algorithm 2.

### 3.5. Embedding with Deep AutoEncoder

We introduce the deep autoencoder (DAE) model to achieve the embedding task. In contrast to the graph embedding methods found in the literature, where road segment vector representation is obtained by aggregating over the neighbouring road segments, our DAE model performs embedding directly on the high-dimensional features of each road segment. As shown in Figure 3, our DAE model comprises three crucial components: the encoder, the embedding space, and the decoder. The encoder component takes the *D*-dimensional road segment feature vectors as input and compresses these into the smaller dimension while preserving as much important information as possible. The preserved *N*-dimensional feature vectors (where *N* ≪ <*D*) are stored in the embedding space. The decoder component aims to reconstruct the original *D*-dimensional road segment features by decompressing the *N*-dimensional features in the embedding space. Taking the above objectives of each component, we can therefore define the learning process of our DAE model into three steps. First, we compress the *D*-dimensional input road segment features (*X*) into *N*-dimensional feature space in the encoder component. Then, we reconstruct the output *Y* from the small dimension using the decoder component. Finally, we calculate the error difference between the original inputs and the reconstructed outputs and adjust the weight parameters to reduce this difference.

Our DAE model is a fully connected network with an input layer, four hidden layers, and an embedding space layer on the encoder component. The decoder component comprises four hidden layers and an output layer. The output layer has the same size as the input layer in the encoder, while the size of the hidden layers in the decoder is similar to the size of the hidden layers in the encoder. We first normalise the road segment feature vectors on the encoder before feeding them to the input layer. Thereafter, we obtain the value of each neuron in the next compressed layer by computing the sum of products of values in the previous layer and their corresponding weight parameters. We then introduce nonlinearities to the network by applying the rectified linear unit (ReLU) activation function defined as ReLU(*x*)=max (0, *x*). On the decoder, we decompress values in the embedding space layer and obtain values in the next decompressed layer using a similar procedure; again, the ReLU function is used as the activation function. Furthermore, we normalise the values in the output layer to be between 0 and 1 through the sigmoid function defined as Sigmoid(*x*)=1/1+*e*^−*x*^. This normalisation is important since input features are also normalised. Finally, we measure the error difference between values in the input layer and their corresponding values in the output layer. Therefore, our optimisation problem is finding the set of optimal weight parameters on the encoder component that achieves the smallest possible error difference. Finally, we extract features in the embedding space layer which we later use to train, validate, and test the machine learning algorithms.  Algorithm 3 shows the step-by-step implementation of our DAE model for an embedding task. The reasons for choosing the number of hidden layers and corresponding sizes will be given in greater detail in Section 4.

The article "Road-Type Classification with Deep AutoEncoder" was published in 2023. Journal: Comput Intell Neurosci.

### 3.6. Road Segment Classification

We use the obtained embedded features, *Z*, in *N*-dimensional feature space (where *N*=8) to compare the performance of deep neural networks (DNN), support vector machines (SVM), and K-nearest neighbors (K-NN) classifiers for road-type classification of road classes mentioned in Section 3.3. These classifiers were chosen for comparison as they are deemed adequate for multiclass classification tasks across various applications [18–23]. Furthermore, these classifiers represent three unique learning methods: the artificial neural networks, the hyperplane-based, and the instance-based learning methods.

The DNN classifier belongs to a family of artificial neural networks where the network's underlying parameters are fine-tuned to match a given class label for each input vector. The SVM is a hyperplane-based learning method that transforms nonlinearly separable input features into a high-dimensional feature space where input features can be separated linearly. The K-NN classifier belongs to the family of instance-based learning methods; unlike the SVM classifier, where two classes are trained simultaneously, the K-NN achieves multiclass classification tasks in one go, where feature vectors (with class labels) representing multiple classes are stored in a feature space. The K parameter is used to decide the class label of the unlabelled vector. Thus, comparing these three classifiers will signify the best learning method for a road-type classification task.

We initially divided the input features into train and test datasets. We perform the 10-fold cross-validation method on the training dataset to obtain optimal parameters for each classifier; then, we use the test dataset to obtain the microaveraged *f*1-score of each classifier based on the optimal parameters.

#### 3.6.1. Deep Neural Networks

The DNN classifier is a fully connected network with the input layer, two or more hidden layers, and the output layer. The size of the input layer corresponds to the number of components (*m*) of road segment feature vectors (*X*=(*x*_*i*_)_*i*=1,2,…,*m*_), and the size of the output layer corresponds to the number of road-type classes (*Y*=(*y*_*i*_)_*i*=1,2,…,*n*_). The size and number of hidden layers are often fine-tuned for optimal results. The embedded road segment features are passed into the input layer; the outputs from the input layer are fed into the 2^*nd*^ layer, the outputs from the 2^*nd*^ layer are fed into the 3^*rd*^ layer, and so on, and ultimately the outputs from the (*L* − 1)^*th*^ layer are fed into the *L*^*th*^ layer; equations (1) and (2) are used to obtain the value of the *i*^*th*^ neuron of the *l*^*th*^ layer, *u*_*i*_^*l*^, by taking the sum of products of values previous layer *l* − 1 and their corresponding weight parameters *W*=(*W*_1_, *W*_2_,…, *W*_*L*_), where *W*_*i*_=(*w*_*i*1_, *w*_*i*2_,…, *w*_*iS*_*i*__), and *S*_*i*_ is the size of the *i*^*th*^ layer.

(1) $$\begin{array}{c} u_{i}^{1}=x_{i},i=1,2,\ldots ,S_{1},S_{1}=m\text{,} \end{array}$$

(2) $$\begin{array}{c} u_{i}^{l}=\overset{S_{l-1}}{\underset{j=0}{\sum }}w_{l-1j}u_{j}^{l-1},i=1,2,\ldots ,S_{l},l=2,3,\ldots ,L\text{,} \end{array}$$

where *w*_*i*0_ is the bias term, *S*_*l*_ is the size of the *l*^*th*^ layer, and *S*_*L*_=*n*.

In equation (3), Sigmoid function, *g*, is applied to compress outputs to be between 0 and 1 and thus obtain probabilities that a given road segment feature vector belongs to a class.

(3) $$\begin{array}{c} v_{i}\left(X,W\right)=g\left(u_{i}^{L}\right),i=1,2,\ldots ,m\text{.} \end{array}$$

Equation (3) determines the predicted class label for each road segment input feature vector *X*. Given a training sample representation (*X*^*k*^, *Y*^*k*^), *k*=1,2,…*N*, such that *Y*^*k*^ determines the class of *X*^*k*^, and *N* is the size of the training sample. The training of our DNN classifier is made by first obtaining the predicted class label, *v*_1_(*X*^*k*^, *W*), *v*_2_(*X*^*k*^, *W*),…, *v*_*n*_(*X*^*k*^, *W*) based on the randomly initialised weight parameters *W* for each road segment vector, *X*^*k*^. The error incurred between predicted outputs and actual class labels *Y*^*k*^=(*y*_1_^*k*^, *y*_2_^*k*^,…, *y*_*n*_^*k*^) for all the training samples is measured by the following formula:

(4) $$\begin{array}{c} E\left(W\right)=\frac{1}{2}\overset{N}{\underset{1}{\sum }}\overset{m}{\underset{j=1}{\sum }}{\left(y_{i}^{k}-v_{i}\left(X^{k},W\right)\right)}^{2}\text{.} \end{array}$$

During the training process, the parameters vector *W* will be updated using the following formula:

(5) $$\begin{array}{c} W=W-\lambda \frac{\partial E}{\partial W}\text{,} \end{array}$$

where *λ* is the learning rate parameter, and *∂E*/*∂W* is the gradient calculated using the backpropagation.  Algorithm 4 shows the steps used to classify road segment features using the DNN classifier.

The article "Road-Type Classification with Deep AutoEncoder" was published in 2023. Journal: Comput Intell Neurosci.

#### 3.6.2. Support Vector Machines

We perform the multiclass road-type classification task using the one vs. one support vector machines (SVM) formulation. In one vs. one SVM, we train two road-type classes at a time; thus, for *M*road-type classes, we obtain a total of *M*(*M* − 1)/2 SVM classifiers; we then assign a class label to the unknown road segment feature vector based on the class with majority counts. For any pair of road-type classes with road segment features from the training dataset and the corresponding class labels (*x*_1_, *y*_1_), (*x*_2_, *y*_2_),…, (*x*_*m*_, *y*_*m*_) and *y* ∈ {−1, +1}, we construct an optimal hyperplane that separates the two classes with the largest possible margin as shown in Figure 4. This margin is defined as the distance between vectors nearest to the optimal hyperplane (support vectors) from both classes.

The *H*_1_ and *H*_2_ planes defined by *wv*_*i*_+*b* ≥ 1 and *wv*_*i*_+*b* ≤ −1 represent the boundaries for feature vectors that belong to two distinct road-type classes. The margin which must then be maximised for the optimal hyperplane is the distance: *d*=2/|*w*| between the *H*_1_ and *H*_2_ planes. We maximize *d* by solving a dual optimisation problem defined as

(6) $$\begin{array}{c} \min\frac{1}{2}w^{2}\text{.} \end{array}$$

Subject to the following constraints:

(7) $$\begin{array}{c} y_{i}=wv_{i}+b\geq 1,\forall i\text{.} \end{array}$$

Furthermore, we introduce Lagrangian's multipliers to eliminate the constraints, and we obtain the dual SVM formulation defined as maximizing

(8) $$\begin{array}{c} L=\underset{i}{\sum }\alpha_{i}-\frac{1}{2}\underset{i}{\sum }\underset{j}{\sum }\alpha_{i}\alpha_{j}y_{i}y_{j}\left(v_{i}\cdot v_{j}\right)\\ subjectto\underset{i}{\sum }\alpha_{i}y_{i}=0,\alpha_{i}\geq 0\text{.} \end{array}$$

Solving the dual SVM yields the coefficients of *α*_*i*_, feature vectors where *α*_*i*_ > 0 are the support vectors, and they lie directly on the *H*_1_ and *H*_2_ planes. The dual SVM problem is 0 for *α*_*i*_=0. Thus, the SVM optimisation problem is affected only by the support vectors. The optimal hyperplane for assigning a class label to an unknown road segment feature vector *v* is done by evaluating the following function:

(9) $$\begin{array}{c} f\left(v\right)=\overset{m}{\underset{i}{\sum }}y_{i}\alpha_{i}\left(x_{i}^{T}\cdot v\right)+b\text{.} \end{array}$$

Radial basis function (RBF) kernel is used to transform nonlinearly separable features to a higher features space *φ* where they can be separated linearly. We compute the transformation by taking the dot product between any pairs of feature vectors using a Kernel function: *K*(*x*_*i*_, *x*{_*j*})=*ϕ*(*x*_*i*_) · *ϕ*(*x*_*j*_). The RBF kernel is defined as follows:

(10) $$\begin{array}{c} K\left(x_{i},x_{j}\right)=\exp\left(\frac{{\left\|x_{i}-x_{j}\right\|}^{2}}{2\sigma^{2}}\right)\text{.} \end{array}$$

Algorithm 5 outlines the steps used to classify road segment features using the SVM classifier.

The article "Road-Type Classification with Deep AutoEncoder" was published in 2023. Journal: Comput Intell Neurosci.

#### 3.6.3. K-Nearest Neighbors

*K*-nearest road segment feature vectors from the training dataset are used to assign a class label to the unknown feature vector. Thus, given road segment features with their corresponding class labels from the training dataset as (*x*_1_, *y*_1_), (*x*_2_, *y*_2_),…, (*x*_*m*_, *y*_*m*_), we calculate the distance between the unknown vector *v* and vectors in the training dataset using the Euclidean distance defined as

(11) $$\begin{array}{c} d\left(u,x_{i}\right)=\sqrt{\overset{m}{\underset{r=1}{\sum }}{\left(c_{r}\left(x_{i}\right)-c_{r}\left(u\right)\right)}^{2}}\text{,} \end{array}$$

where *c*_*r*_(*u*) is the value of the *r*^*th*^ component of the vector *u*.

We then define a set *V*={*v*_1_, *v*_2_ …, *v*_*K*_} of *K* features from the training dataset nearest to the unknown feature to assign its class label. According to equation (12), the unknown feature vector *u* is assigned to a class that appears the most within a set of *K*-nearest feature vectors.

(12) $$\begin{array}{c} l_{u}⟵\underset{v\in V}{\mathrm{argmax}}\overset{K}{\underset{i=1}{\sum }}\delta \left.\left(l_{v},y_{i}\right)\right)\text{,} \end{array}$$

where *y*_*i*_ is the class of sample *x*_*i*_, *l*_*v*_ is the class label of the vector *v*, and the function *δ* is defined as follows:

(13) $$\begin{array}{c} \delta \left(x,y\right)=\left\{\begin{array}{cc} 1\text{,} & \text{if}\;x=y\text{,}\\ 0\text{,} & \text{otherwise}. \end{array}\right. \end{array}$$

Algorithm 6 lists the steps used to classify road segment features using the K-NN classifier. Inputs are the feature vectors initially divided into training and test datasets. We use the training dataset to train the classifier and obtain the optimal *K* through cross-validation. We use the test dataset to obtain the accuracy of the K-NN classifier based on the optimal *K* value.

The article "Road-Type Classification with Deep AutoEncoder" was published in 2023. Journal: Comput Intell Neurosci.

## 4. Experimental Results and Discussion

The Linkoping city road networks graph dataset [24] is used to train our DAE embedding method. Embedded features are used to train, validate, test, and compare DNN, SVM, and K-NN classifiers for road segment classification tasks. Classifier with the highest microaveraged *f*1-score is selected, and results achieved are compared to some state-of-the-art embedding methods found in the literature for solving a similar problem. Experiments are designed mainly to obtain optimal parameters on our DAE embedding method and classifiers.

### 4.1. Embedding with Deep AutoEncoder

Input to our DAE embedding method is a total of 6761, and 58-dimensional road segment feature vectors described in Section 3.3. First, the dataset is divided into a 70/30 split, where 70% of the dataset is used to train the DAE model while the remaining portion of the dataset obtains optimal parameters of the DAE method. Optimisation is achieved through the Adam optimiser, while the batch size and maximum iterations were chosen as 1024 and 500, respectively. As depicted in Table 3, we define several DAE models with varying numbers of hidden layers and sizes on the encoder and decoder component and the layer size on the embedding space. This is done to identify optimal parameters that achieve the lowest reconstruction error and the highest accuracy using the validation dataset.

We train each DAE model listed in Table 3 using different learning rates {1*e*^−4^, 1*e*^−3^, 1*e*^−2^}, and we report the results in terms of the reconstruction error and accuracy based on the validation dataset after 500 iterations. We then select the DAE model with a corresponding learning rate that achieves the lowest average reconstruction error and the highest accuracy as our optimal DAE embedding method.

The article "Road-Type Classification with Deep AutoEncoder" was published in 2023. Journal: Comput Intell Neurosci.

Figures 5–7 show the performances of three DAE models at increasing learning rates in terms of reconstruction error and validation accuracy. It can be observed that the DAE model with 5 hidden layers and embedding space of 4 units achieved the lowest reconstruction error and the highest accuracy of 0.0013 and 98.82%, respectively, at a learning rate of 1*e*^−3^. The DAE model with 4 hidden layers and embedding space of 8 units achieved the lowest reconstruction error and the highest accuracy of 0.000578 and 99.11%, respectively, at a learning rate of 1*e*^−3^. Finally, the DAE model with 3 hidden layers and embedding space of 10 units achieved the lowest reconstruction error and the highest accuracy of 0.000623 and 98.96%, respectively, at a learning rate of 1*e*^−3^. Based on these observations, we select our DAE embedding method using the model with 4 hidden layers and embedding space of 8 units as it achieves better performance.

### 4.2. Road-Type Classification

Input dataset to the DNN, SVM, and K-NN classifiers is 6761 road segment features of 8 dimensions obtained by our DAE embedding method. The dataset comprises 5 classes of merged and relabelled road types according to the method described in Section 3.3. We initially divided the dataset into a 70/30 split, where 70% of the data are used to train and validate the classifiers based on the 10-foldcross-validation method. We use the remaining 30% of the data to test the classifiers' performance in the microaveraged *f*1-score based on the optimal parameters obtained by the 10-foldcross-validation method. We obtain the micro *f*1-score of each classifier by first computing the confusion matrix; thereafter, we calculate the sums of the true positives (TP), false positives (FP), and false negatives (FN) across all the classes.

#### 4.2.1. Classification with DNN

Road-type classification with DNN was achieved using the steps mentioned in Algorithm 4. Optimisation was performed using the Adam optimiser, and the ReLU function as the activation function. Various learning rates and the number of hidden layers and sizes were investigated to identify the optimal parameters. The number of hidden layers and sizes was as follows: Layers *A* = {64, 128, 64}, Layers *B* = {64, 128, 128, 64}, Layers *C* = {400, 800, 800, 400}, and Layers *D* = {300, 500, 800, 800, 500, 300}. Through the 10-foldcross-validation method, we obtained optimal learning rate of *u*=0.001 and six hidden layers (Layers *D*), respectively, as indicated in Table 4.

We used the obtained optimal parameters to train and test the DNN classifier, and we report the results obtained from the test dataset using the microaverage *f*1-score shown in Table 5.

The article "Road-Type Classification with Deep AutoEncoder" was published in 2023. Journal: Comput Intell Neurosci.

#### 4.2.2. Classification with SVM

Road-type classification with SVM was achieved using the steps mentioned in Algorithm 5. The one vs. one SVM formulation was used, thus giving a total of 10 classifiers. Through the 10-foldcross-validation method, we obtained optimal RBF kernel width of *σ*=5 and the error term parameter of *c*=100 as indicated in Table 6.

We then used the obtained optimal parameters to train and test the SVM classifier; we report the results obtained from the test dataset using the microaverage *f*1-score as shown in Table 7.

#### 4.2.3. Classification with K-NN

Road-type classification with K-NN was performed using the steps mentioned in Algorithm 6. Through the 10-foldcross-validation method, we obtained the optimal K value of 5 as shown in Table 8.

We used the obtained optimal parameter to train and test the K-NN classifier, and we report the results obtained from the test dataset using the microaverage *f*1-score as shown in Table 9.

Tables 5–7 show the performances of three classifiers using microaveraged *f*1-score for road segment classification tasks. It can be observed that the DNN is the best-performing classifier with the micro *f*1-score of 80.16%. The second best performing classifier is the K-NN, with the micro *f*1-score of 76.13%. The SVM is the worst-performing classifier with the micro *f*1-score of 70.98%.

### 4.3. Comparison to Other Methods

We then compared the highest microaveraged *f*1-score obtained by our DAE model with some of the state-of-the-art embedding methods presented in [2] for the road-type classification task. Some of the similarities between our study and the study proposed in [2] are as follows: both studies were carried out using the Linkoping City road network graph dataset extracted from OSMnx, both studies transform the original graph to line graph to obtain more descriptive features for each road segment, and both studies similarly construct a 58-dimensional feature vector representing each road segment. Training of embedding methods for both studies is achieved using 500 iterations and 1024 batch size while optimisation is achieved using the Adam optimiser. The major difference between the two studies is how embedding is achieved. Our DAE method achieves embedding by reducing the dimensionality of each road segment feature vector, while the methods proposed in [2] achieve embedding on each road segment vector by aggregating information from its neighbouring road segments. The final embedded vector obtained from our DAE method has 8 dimensions, while the methods proposed in [2] have the final embedded vectors obtained from one of the output dimensions {64,128,56}.

The article "Road-Type Classification with Deep AutoEncoder" was published in 2023. Journal: Comput Intell Neurosci.

Table 10 shows the comparison of the performance of the methods in terms of the micro *f*1-score. Our DAE embedding method achieves the micro *f*1-score of more than 20% when compared to raw features (original 58-dimensional features without embedding). Furthermore, our DAE method outperforms the GCN, GSAGE-MEAN, GAT, and GIN methods by micro *f*1-score of 22%, 18%, 5%, and 2%, respectively. We also observe that our DAE method achieves the same micro *f*1-score of 80% as the GSAGE-MAXPOOL method. Finally, our DAE methods fall short by micro *f*1-score of 1% compared to the GSAGE-MEANPOOL and GAIN methods.

One of the reasons why the proposed method outperforms the state-of-the-art graph embedding methods is that the two methods perform embedding differently. Our DAE acknowledges that not all 58 features representing each road segment are necessary; thus, it performs embedding by reducing the dimensionality of each road segment from 58 dimensions to 8 dimensions representing the most prominent features. On the graph embedding methods, embedding on each road segment feature vector is performed by using the feature vectors of neighbouring road segments; while this allows for modelling spatial connection of road segments, the fact that some features in each road segment are not necessary is ignored, thus yielding less performance compared to our DAE method.

## 5. Discussion

This study presents a novel representation learning method for a road-type classification task. Compared to other methods found in the literature, which normally perform embedding on each road segment by aggregating information from neighbouring road segments, our method performs embedding by reducing the dimensionality of each road segment while preserving only the important features using the deep autoencoder (DAE) model. To compare the methods fairly, we conducted our experiments using the Linkoping city road networks graph dataset extracted from OSMnx. We then used the same line graph transformation and feature engineering methods as in [2] to represent road segments as nodes and obtain more descriptive features of each road segment, respectively. We then passed the road segment vectors to our DAE embedding methods, obtaining more robust features at much smaller dimensions than the original ones.

We then passed the vectors obtained by our DAE embedding method to the deep neural networks (DNN), support vector machines (SVM), and K-nearest neighbor classifier (K-NN) classifiers to select best performing classifier using the microaveraged *f*1-score. As shown in Tables 5–9, we demonstrated that the DNN is the best performing classifier for road-type classification task of the vectors obtained by our DAE method. We compared our DAE method to some of the state-of-the-art methods experimented in [2] for solving a similar task. These methods include graph convolution networks (GCN), GraphSAGE (MEAN, MEANPOOL, MAXPOOL, and LSTM), graph attention networks (GAT), graph isomorphism networks (GIN), and graph attention isomorphism networks (GAIN).

The article "Road-Type Classification with Deep AutoEncoder" was published in 2023. Journal: Comput Intell Neurosci.

In Table 10, we demonstrated that our method outperforms the GCN, GSAGE-MEAN, GAT, and GIN methods while achieving similar performance to GSAGE-MAXPOOPL. Furthermore, we observed that our method falls short by 1%, compared to the GSAGE-MEANPOOL and GAIN methods. It is worth mentioning that GSAGE-MEANPOOL and GAIN embedding methods achieve the best performances at much larger dimensions of the embedded feature vectors compared to our method, which achieves comparable performance at a much smaller dimension of the embedded vectors. We also note from Tables 5–9 that merging and relabelling different road types using the method shown in Table 1 is not ideal as several classes (class 2 and class 3) are characterised by many false negatives across all three classifiers, thus, resulting in low micro *f*1-score in all classifiers.

## 6. Conclusion

This paper proposes a novel deep autoencoder (DAE) embedding method for road-type classification tasks. We used the state-of-the-art feature extraction method found in the literature and represented each road segment as a feature vector. We then applied our DAE embedding method and obtained embedded road segment features which we later used to train, validate, and test several machine learning classifiers. We compared our results to several state-of-the-art graph embedding methods and demonstrated that our method outperforms some of these methods while achieving comparable results to others. It is worth noting that our method performs embedding by reducing the dimensionality of each road segment vector. In contrast, the graph embedding methods in the literature achieve road segment embedding using the neighbouring road segment features. Therefore, future work will employ a double embedding technique where the vectors obtained by our DAE method are fed as inputs to the graph embedding methods proposed in the literature.

## Figures and Tables

**Figure 1:** System diagram of the proposed method.

**Figure 2:** Line graph transformation: edges in the original graph are nodes in the transformed graph, and edges that share a node in the original graph become an edge in the transformed graph.

**Figure 3:** Illustration of the basic deep autoencoder model.

**Figure 4:** Application of the SVM classifier on two road-type classes.

**Figure 5:** Performance of DAE model at 5 hidden layers of size {49, 40, 31, 22, 13} on the encoder and decoder; and embedding space of size 4: (a) reconstruction error at increasing learning rates and (b) validation accuracy at increasing learning rates.

The article "Road-Type Classification with Deep AutoEncoder" was published in 2023. Journal: Comput Intell Neurosci.

**Figure 6:** Performance of DAE model at 4 hidden layers of size {48, 38, 28, 18} on the encoder and decoder; and embedding space of size 8: (a) reconstruction error at increasing learning rates and (b) validation accuracy at increasing learning rates.

**Figure 7:** Performance of DAE model at 3 hidden layers of size {46, 34, 22} on the encoder and decoder; and embedding space of size 10: (a) reconstruction error at increasing learning rates and (b) validation accuracy at increasing learning rates.

**Algorithm 1:** Line graph transformation.

**Algorithm 2:** Feature generation for each road segment.

**Algorithm 3:** Feature embedding with deep autoencoder.

**Algorithm 4:** Road segment classification using DNN.

**Algorithm 5:** Road segment classification using SVM.

**Algorithm 6:** Road segment classification using K-NN.

**Table 1:** Merged and relabelled road types.

Class	Merged road labels	Nodes count
Class 1	Highway, yes, primary, secondary, motorway-link, trunk-link, primary-link, secondary-link	1140
Class 2	tertiary, tertiary-link	951
Class 3	Road, planned, unclassified	922
Class 4	Residential	3012
Class 5	Living street	736

**Table 2:** Road segment feature generation.

Graph	Road segment attributes	Dimension
*G*	Road segment length	1-dimension
*L*(*G*)	Midpoint coordinates between two nodes in longitude and latitude	2-dimensions
*L*(*G*)	Subtraction of 20 equally spaced distanced points by the midpoint coordinates	40-dimensions
*G*	One hot encoding of speed limit	15-dimensions

**Table 3:** Hyperparameter settings for optimal DAE parameters.

No. of hidden layers	Layer size		
	Encoder	Embedding space	Decoder
5	{58, 49, 40, 31, 22, 13}	4	{13, 22, 31, 40, 49, 58}
4	{58, 48, 38, 28, 18}	8	{18, 28, 38, 48, 58}
3	{58, 46, 34, 22}	10	{22, 34, 46, 58}

**Table 4:** Average micro *f*1-score for DNN classifier across 10-fold CV at layers and *u* parameters.

*u*=0.0001		*u*=0.001		*u*=0.01	
Hidden layer size	Avg. micro *f*1-score	Hidden layer size	Avg. micro *f*1-score	Hidden layer size	Avg. micro *f*1-score
Layers A	0.67	Layers A	0.77	Layers A	0.74
Layers B	0.71	Layers B	0.77	Layers B	0.69
Layers C	0.71	Layers C	0.79	Layers C	0.76
Layers D	0.74	**Layers D**	**0.81**	Layers D	0.78

Bold values indicate optimal DNN classifier parameters (hidden layers and learning rate) and the corresponding micro averaged *f*1-score.

**Table 5:** Micro *f*1-score for DNN classifier at optimal parameters.

Class	TP	FN	FP	Micro *f*1-score
Class 1	279	63	55	*f*1=*TP*/*TP*+1/2(*TP*+*FN*)*∗*100=80.16%
Class 2	162	123	73	
Class 3	201	76	85	
Class 4	811	93	145	
Class 5	172	49	42	
Total	1625	404	400	

The article "Road-Type Classification with Deep AutoEncoder" was published in 2023. Journal: Comput Intell Neurosci.

**Table 6:** Average micro *f*1-score for SVM classifier across 10-fold CV at *c* and *σ* parameters.

*c* = 1		*c* = 10		*c* = 100	
Sigma: *σ*	Avg. micro *f*1-score	Sigma: *σ*	Avg. micro *f*1-score	Sigma: *σ*	Avg. micro *f*1-score
0.0001	0.43	0.0001	0.55	0.0001	0.57
0.01	0.57	0.01	0.57	0.01	0.62
0.2	0.62	0.2	10.62	0.2	0.65
2	0.62	2	0.64	2	0.67
5	0.62	5	0.63	**5**	**0.69**

Bold values indicate optimal SVM classifier parameters (sigma and error term) and the corresponding micro averaged *f*1-score.

**Table 7:** Micro *f*1-score for SVM classifier at optimal parameters.

Class	TP	FN	FP	Micro *f*1-score
Class 1	301	41	113	*f*1=TP/TP+1/2(TP+FN)*∗*100=70.98%
Class 2	150	135	91	
Class 3	128	149	49	
Class 4	851	53	326	
Class 5	16	205	20	
Total	1446	583	599	

**Table 8:** Average micro *f*1-score for K-NN classifier across 10-fold CV at each *K* parameter.

*K* Parameter	Avg. micro *f*1-score
1	0.73
3	0.74
**5**	**0.76**
7	0.75
9	0.74
11	0.74

Bold values indicate optimal KNN classifier parameter (K value) and the corresponding micro averaged *f*1-score.

**Table 9:** Micro *f*1-score for K-NN classifier at optimal parameters.

Class	TP	FN	FP	Micro *f*1-score
Class 1	309	33	108	*f*1=TP/TP+1/2(TP+FN)*∗*100=76.31%
Class 2	155	130	81	
Class 3	169	108	66	
Class 4	749	155	144	
Class 5	166	55	81	
Total	1548	481	480	

**Table 10:** Method comparisons using micro *f*1-score.

Method	Micro *f*1-score (%)
Raw features [2]	59
GCN [2]	58
GSAGE-MEAN [2]	62
GSAGE-MEANPOOL [2]	81
GSAGE-MAXPOOL [2]	80
GSAGE-LSTM [2]	81
GAT [2]	75
GIN [2]	78
GAIN [2]	81
**DAE (proposed)**	**80**

Bold values indicate the micro averaged *f*1-score obtained by our proposed method (DAE).

## Data Availability

The datasets analyzed during the current study are available at https://planet.openstreetmap.org/.
